The article "Expression of carbonic anhydrase 9, a potential intrinsic marker of hypoxia, is associated with poor prognosis in oesophageal squamous cell carcinoma" was published in 2008. Journal: Br J Cancer.

# Expression of carbonic anhydrase 9, a potential intrinsic marker of hypoxia, is associated with poor prognosis in oesophageal squamous cell carcinoma

**DOI:** 10.1038/sj.bjc.6604719

**Published:** 2008-10-07

**Authors:** N Tanaka, H Kato, T Inose, H Kimura, A Faried, M Sohda, M Nakajima, Y Fukai, T Miyazaki, N Masuda, M Fukuchi, H Kuwano

**Affiliations:** 1 Department of General Surgical Science, Gunma University, Graduate School of Medicine, Maebashi, Japan

**Keywords:** carbonic anhydrase 9, hypoxia, prognosis, oesophageal squamous cell carcinoma

## Abstract

Carbonic anhydrase 9 (CA9) is a protein to be upregulated under exposure to hypoxic conditions. Hypoxic conditions are known to be associated with resistance to chemotherapy and radiotherapy, and with poor cancer prognosis. We examined CA9 expression in surgical specimens from oesophageal squamous cell carcinoma (ESCC) patients (*n*=127) using immunohistochemistry and real-time RT–PCR. We also examined CA9 expression and cell proliferation in ESCC cell lines (TE-2, TE-8 and TE-15) and an immortalised human oesophageal cell line (CHEK-1) using real-time RT–PCR, Western blotting, ELISA and MTT assay. Immunohistochemistry, high expression of CA9 was found in 63 of the 127 primary tumour specimens and was correlated with poor outcome (*P*=0.0003) and more aggressive/less favourable clinicopathological parameters (tumour size (*P=*0.0235), tumour depth (*P*<0.0001), regional lymph node metastasis (*P=*0.0031), distant lymph node metastasis (*P=*0.0077), stage (*P*<0.0001) and blood vessel invasion (*P=*0.006)). *In vitro*, CA9 expression in cultured cells and culture medium was also induced by hypoxia (*P*<0.01). CA9 is correlated with poor prognosis and malignant phenotype in patients with ESCC, and was upregulated by hypoxia. It is suggested that control of CA9 expression might improve the effectiveness of chemotherapy and radiotherapy in ESCC.

Oesophageal cancer is a common malignant neoplasm throughout the world. Despite recent improvements in surgical techniques, chemotherapy and radiation treatment, the prognosis for patients with advanced disease is still unsatisfactory (Collard *et al*, 2001; Ando *et al*, 2003). New approaches to increase the effectiveness of chemotherapy and radiotherapy need to be developed to improve the prognosis of oesophageal cancer.

A hypoxia tumour environment is known to be associated with resistance to chemotherapy and radiotherapy, and with more malignant tumour phenotypes that show increased invasiveness, greater metastatic potential and poor survival (Gray *et al*, 1953; Brizel *et al*, 1996; Hockel *et al*, 1996). Clinical studies have shown a strong correlation between low pretreatment tumour pO_2_ and poor tumour control and overall survival in patients with head and neck squamous cell carcinoma (Brizel *et al*, 1999; Nordsmark *et al*, 2003).

Carbonic anhydrase 9 (CA9), such as hypoxia-inducible factor 1α (HIF-1α), is known to be a marker of hypoxia, but its role in a hypoxic tumour microenvironment is still unclear (Wykoff *et al*, 2000). The carbonic anhydrase (CA) family of zinc metalloenzymes include at least 14 different isoforms in mammals. Some of these isozymes are cytosolic (CA1, CA2, CA3, CA7, CA13) and others are membrane-bound (CA4, CA9, CA12 and CA14), whereas CA 5 is mitochondrial and CA6 is secreted into saliva and milk. Three cytosolic acatalytic forms are also known (CARP8, CARP10 and CARP11) (Pastorekova *et al*, 2004). CA is involved in the reversible hydration–dehydration of carbon dioxide, CO_2_+H_2_O↔HCO_3_^−^+H^+^. The CA family plays a variety of roles in many physiologic processes, including pH regulation and maintenance of ionic equilibrium (Maren, 1967; Tashian, 1989). Two of the carbonic anhydrases, CA9 and CA12, are transmembrane isozymes that are highly expressed in some tumours, and may be implicated in acidification of the extracellular milieu surrounding cancer cells, thus creating a microenvironment conducive to tumour growth and spread (Pastorek *et al*, 1994; Ivanov *et al*, 1998; Türeci *et al*, 1998; Parkkila *et al*, 2000).

CA9 expression has been associated with poor prognosis in patients with lung, breast, cervical, brain, and renal cancer (Chia *et al*, 2001; Giatromanolaki *et al*, 2001; Loncaster *et al*, 2001; Bui *et al*, 2003; Brennan *et al*, 2006; Haapasalo *et al*, 2006) and with resistance to chemotherapy in head and neck cancers (Koukourakis *et al*, 2001). It has been reported that CA9 expression is an independent prognostic marker in oesophageal and gastric adenocarcinomas (Driessen *et al*, 2006), but the relationship between prognosis and CA9 expression in oesophageal squamous cell carcinoma (ESCC) remains controversial. *In vitro* studies have indicated that CA9 plays a role in the growth and survival of breast carcinoma cells (Robertson *et al*, 2004); but its precise function in normal and cancerous tissues remains unclear.

The purpose of this study was to investigate CA9 expression in patients with ESCC, and to confirm changes in the expression level of CA9 in ESCC cell lines and culture medium under hypoxic conditions.

## Materials and methods

### Clinical samples

This study was performed on 127 patients with ESCC who underwent potentially curative surgery without preoperative therapy at the Department of General Surgical Science, Gunma University Graduate School of Medicine, between 1983 and 2004. Tumour stage was classified according to the sixth edition of the tumour-node-metastasis classification of the International Union against Cancer (UICC) (Sobin and Witteking, 2002). All patients signed informed consent forms in accordance with our institutional guidelines. Information on gender, age, stage of disease, and histopathologic factors was abstracted from medical records.

Before analysis, the resected specimens were fixed with 10% formaldehyde, embedded in paraffin blocks, cut into 4-*μ*m thick sections, and mounted on glass slides. Paraffin-embedded sections were acquired from all 127 patients (112 males and 15 females). The median age of these patients was 62 years (range, 40–79 years), and the median survival time was 30.2 months (range, 1–220 months).

### Immunohistochemistry

Immunohistochemical staining of the sections for CA9 expression was performed using the standard streptavidin–biotin peroxidase complex method, as described earlier (Kato *et al*, 2002; Fukai *et al*, 2005). Each 4-*μ*m thick section was deparaffinised, rehydrated and incubated with fresh 0.3% H_2_O_2_ in methanol for 30 min at room temperature to block endogenous peroxidase activity. After rehydration through a graded series of ethanol concentrations, the sections were autoclaved in 10 mM citrate buffer (pH 6.0) at 120°C for 3 min, and then cooled to 30°C. After rinsing in 0.1 M phosphate-buffered saline (PBS; pH 7.4), non-specific binding sites were blocked by incubation with 10% normal goat serum for 30 min. The sections were then incubated at 4°C overnight with a rabbit polyclonal antibody (Novus Biologicals Inc., Littleton, USA) at a dilution of 1 : 2500 in PBS containing 1% bovine serum albumin. The sections were then washed in PBS, incubated with biotinylated anti-rabbit IgG for 30 min at room temperature, and finally incubated in streptavidin–biotin peroxidase complex solution (Nichirei Co., Tokyo, Japan). The chromogen, 3,3′-diaminobenzidine tetrahydrochloride, was applied as a 0.02% solution containing 0.005% H_2_O_2_ in 50 mM ammonium acetate–citrate acid buffer (pH 6.0). Finally, the sections were lightly counterstained with Mayer’s haematoxylin and mounted. Normal gastric mucosa served as a positive control.

### Scoring of CA9 protein expression

CA9 expression was evaluated by calculating an immunostaining score, which was the product of the intensity score and the staining rate. Only membranous staining was considered positive. We evaluated tumours at their surface (*n*=121), centre (*n*=127) and invasive front (*n*=125). In accordance with the reported criteria (Chia *et al*, 2001; Driessen *et al*, 2006), the intensity score was based on the estimated staining intensity (0, no staining (Figure 1A); 1, weak (Figure 1B); 2, moderate (Figure 1C); 3, strong (Figure 1D)), and the staining rate was defined as the percentage of tumour cells that showed positive staining for CA9 (0–100%). The final immunostaining score (IHC score: 0–300) was calculated as the product of the staining intensity and the staining rate for each CA9-positive tumour. The tumours were considered to have high CA9 expression if the final score exceeded the median score (Driessen *et al*, 2006).

### RNA isolation and cDNA synthesis

Total RNA was extracted from fresh-frozen sections and cell lines using an RNeasy Mini kit (Qiagen, Hilden, Germany) in accordance with the manufacturer’s instructions. Clinical fresh-frozen sections were taken from peripheral tumour areas. The quantity of isolated RNA was measured using an ND-1000 spectrophotometer (NanoDrop Technologies, Wilmington, Delaware). Template cDNA was synthesised from 13.5 *μ*g of total RNA using an Omniscript Reverse Transcriptase kit (Qiagen), random primer (hexadeoxyribonucleotide mixture) (TaKaRa, Shiga, Japan) and ribonuclease inhibitor (Porcine liver) (TaKaRa). Total RNA was reverse-transcribed with four units of Omniscript Reverse Transcriptase in a reaction volume of 20 *μ*l (60 min at 37°C, 5 min at 93°C, and finally on ice). The resulting cDNA samples were stored at −30°C until analysis.

### Real-time reverse transcriptase–polymerase chain reaction

Real-time reverse transcriptase (RT)–PCR analyses were performed on an ABI Prism 7000 Sequence detection system (Applied Biosystems, Foster City, CA, USA). The standard reaction volume was 20 *μ*l and contained 1 × SYBR Green PCR Master Mix (ABI), 2.0 *μ*l of cDNA template, and both forward and reverse primers at 10 *μ*M. The initial PCR denaturation step was performed for 5 min at 95°C, followed by 40 cycles of 60 s at 95°C (melting) and 60 s at 60°C (annealing/elongation). All reactions were performed in duplicate. The data were normalised to an internal control gene, *β*-actin, to control for the amount of RNA in the preparation.

### Oligonucleotide primers for CA9 gene amplification by RT–PCR

The oligoribonucleotide primers for CA9 were sense primer 5′-CCTCAAGAACCCCAGAATAATGC-3′; antisense primer 5′-CCTCCATAGCGCCAATGACT-3′, and those for *β*-actin were: sense primer 5′-CTCCTCCTGAGCGCAAGTACTC-3′; antisense primer 5′-TCCTGCTTGCTGATCCACATC-3′. The amplification was performed for 30 cycles of 30 s at 94°C, 30 s at 62°C (55°C for *β*-actin) and 30 s at 72°C. Primers for CA9 and *β*-actin were used with reference to previously published assays (Furuya *et al*, 2004; Simi *et al*, 2006).

### Cell lines

Three human ESCC cell lines and one immortalised human oesophageal cell line were used: TE-2, TE-8, TE-15 and immortalised human oesophageal cell line (CHEK-1), respectively. TE-2, TE-8 and TE-15 were kindly provided by Dr T Nishihira, Institute of Development, Aging and Cancer, Tohoku University School of Medicine, Sendai, Japan. CHEK-1 cells were kindly provided by Dr H Matsubara. CHEK-1 was established by transfection of human papillomavirus type 16 E6/E7 into primary cultures of human oesophageal keratinocytes (Sashiyama *et al*, 2002). All cancer cell lines were derived from ESCC with varying degrees of differentiation (Nishihira *et al*, 1993). TE cell lines and CHEK-1 cells were cultured in RPMI-1640 medium (Sigma Chemical Co., St Louis, MO, USA) supplemented with 10% fetal bovine serum and antibiotics (100 U ml^−1^ penicillin and 100 *μ*g ml^−1^ streptomycin). All cell lines were cultured to 70–80% confluence.

Parallel incubation was performed on aliquots of cells under normoxic (humidified air with 5% CO_2_) and hypoxic conditions. Hypoxic conditions were generated in the APM-30D incubator (ASTEC Inc., Fukuoka, Japan) with 1% O_2_, 5% CO_2_ and balance N_2_, after incubation in normoxic conditions for 24 h.

### Western blot analysis

Lysates from exponentially growing cell lines were prepared in buffer (20 mM Tris-HCl, pH 7.6, 1 mM EDTA, 140 mM NaCl, 1% Nonidet P-40, 1% aprotinin, 1 mM phenylmethylsulphonyl fluoride and 1 mM sodium vanadate). The protein concentration was determined using a BCA Protein Assay Kit (Pierce, Rockford, IL, USA). Protein (40 *μ*g) from each cell line was resuspended in a sodium dodecyl sulphate (SDS) sample buffer (100 mM Tris-HCl, pH 8.8, 0.01% bromophenol blue, 36% glycerol and 4% SDS) containing 1 mM dithiothreitol, boiled for 10 min and applied to a 5–20% gradient Ready-Gel (Bio-Rad, Tokyo, Japan). Proteins were electrotransferred to a Hybond-enhanced chemiluminescence nitrocellulose membrane (Amersham Pharmacia Biotech, Buckinghamshire, UK). Proteins were immunoblotted using anti-CA9 (Novus Biologicals Inc.) The bands were detected using the enhanced chemiluminescence detection system (Amersham Pharmacia Biotech). For re-blotting, membranes were stripped according to the manufacturer’s protocol. An anti-*β*-actin antibody (Sigma Chemical Co.) served as a control. Horizontal scanning densitometry was performed using acquisition into Adobe Photoshop (Apple Inc., Cupertino, CA, USA) and results were analysed by Quantity One (Bio-Rad).

### ELISA

The CA9 concentration in the cell culture supernatants was determined by ELISA using a Quantikine® Human Carbonic Anhydrase IX/CA9 Immunoassay Kit (R&D Systems, Minneapolis, MN, USA) in accordance with the manufacturer’s instructions. The samples were collected from supernatants of cell lines that had been cultured under normoxic and hypoxic conditions. After centrifugation at 1500 r.p.m., the samples were thawed at 4°C overnight. Then, 50 *μ*l of buffered protein base and 100 *μ*l of sample were added to the wells of a microtitre plate coated with an anti-CA9 mouse monoclonal antibody and incubated for 2 h at room temperature on a horizontal orbital microplate shaker. The plate was washed four times, and 200 *μ*l of conjugated antibody solution was then added. After further incubation, the plate was washed again, 200 *μ*l of substrate solution was added, and a third incubation was carried out for 30 min at room temperature, with protection from light. After the addition of 50 *μ*l of stop solution, colour development was determined immediately at 450 nm using a microtitre plate reader. All samples were assayed three times in a blinded manner, and the mean was used for data analysis.

### *In vitro* proliferation assay

Cell proliferation was measured in ESCC cells using the MTT tetrazolium assay. Briefly, ESCC cells (2.5 × 10^3^ per well) were plated in 96-well plates, 100 *μ*l for each well. After initial cell seeding, the WST-1 assay (Dojin, Tokyo, Japan) was performed, and 10 *μ*l of the cell counting solution was added to each well of the plates, followed by incubation in a humidified 5% CO_2_ atmosphere at 37°C for 3 h. The formazan was dissolved in 90 *μ*l per well 1 N HCl, and the absorbance of the solution was read at 450 nm using a microtitre plate reader (Becton Dickinson, Franklin Lakes, NJ, USA). All experiments were performed in triplicate.

### Statistical analysis

Statistical analysis was performed using the *χ*^2^ test, Fisher’s exact test and Mann–Whitney *U*-test. Survival curves were calculated by the Kaplan–Meier method and analysis was carried out using the log-rank test. Prognostic factors were examined by univariate and multivariate analyses using a Cox proportional hazards model. Differences at *P*<0.05 were considered significant. For statistical analyses, we used Stat View Version 5.0 software (SAS Institute Inc., Cary, NC, USA).

## Results

### Clinical samples

#### Expression of CA9 protein in ESCC

Staining for CA9 in the normal oesophageal squamous epithelium was negative (Figure 1A), but it was clearly positive in the gastric mucosa used as a positive control (Figure 1A). In cancer cells, CA9 staining was seen mainly in the plasma membrane, and at the border of tumours only the cancerous lesion showed positive staining (Figure 1B–D). In the tumour centre, 76 (59.8%) of the 127 primary tumour specimens showed CA9 positivity. In the tumour surface, 39 (32.2%) of the 121 primary tumour specimens showed CA9 positivity, whereas in the tumour-invasive front, 28 (22.4%) of 125 primary tumour specimens showed CA9 positivity.

#### Correlations between CA9 expression and clinicopathological findings

For examination of the tumour centre, we divided the tissue sections into a high group and a low group, on the basis of their IHC scores (range, 0–250.2; median, 12.8; mean, 46.7). A median immunostaining score >12.8 was considered to indicate high CA9 expression. Sixty-three of the 127 patients were classified in the high CA9 expression group and the other 64 patients were classified in the low expression group. This classification was in agreement with earlier reports (Chia *et al*, 2001; Driessen *et al*, 2006). The correlation between the clinicopathologic characteristics of the ESCC patients and tumour centre CA9 expression is summarised in Table 1. CA9 expression was correlated with tumour size (*P=*0.0235), tumour depth (*P*<0.0001), regional lymph node metastasis (*P=*0.0031), distant lymph node metastasis (*P=*0.0077), stage (*P*<0.0001) and blood vessel invasion (*P=*0.006). However, there was no significant association between CA9 expression and other factors, such as age, gender, histological differentiation, tumour location and lymphatic invasion. We did scoring for all three parts (tumour surface, tumour centre and invasive front) using the method that we described in the paper. There were no associations between the relevant clinicopathological parameters and CA9 staining assessed at the tumour surface or invasive front.

#### Prognostic significance of CA9 expression

The survival rate of patients with tumours showing low CA9 expression was significantly higher than that of patients with tumours showing high CA9 expression (*P*=0.0003; Figure 2). The 5-year survival rate for patients with low CA9 expression was significantly higher than that of patients with high CA9 expression (66.5 *vs* 33.3%). In univariate Cox proportional hazards analysis, primary tumour (T), regional lymph node metastasis (N), distant metastasis (M), TNM stage (S) and CA9 expression were the strongest prognostic factors for cancer-specific survival. However, tumour CA9 expression in ESCC patients was not identified as an independent prognostic factor in multivariate survival analysis using Cox proportional hazards analysis (Table 2).

#### CA9 mRNA expression determined by real-time RT–PCR

To confirm CA9 mRNA expression, we analysed 35 clinical samples, including normal and tumour tissue. All samples quantified values used to calculate CA9/*β*-actin expression ratios. In this group of paired samples, CA9 mRNA expression levels were significantly higher in tumour tissues (0.022±0.038) (mean±s.d.) than in normal tissues (0.009±0.016). This resulted in a significant difference in the mRNA expression level between tumour and normal tissues (*P*=0.0019; Figure 3).

### Cell lines

#### Expression of CA9 mRNA cell lines during normoxia and hypoxia

We initially investigated the mechanism of CA9 regulation in ESCC during hypoxia by examining mRNA expression. We cultured the cell lines TE-2, TE-8 and TE-15 for 24 h under hypoxic conditions (1% O_2_). We then compared CA9 mRNA levels between hypoxic and normoxic conditions using RT–PCR. In all three cell lines, expression of CA9 mRNA was upregulated under hypoxic conditions (Figure 4).

#### Expression of CA9 in ESCC cell line TE-2 under hypoxic conditions

We compared the temporal expression of CA9 mRNA in the ESCC cell line TE-2 and in the CHEK-1 under hypoxic conditions. In TE-2 cells, the ratio between CA9 mRNA expression during hypoxia relative to normoxia increased markedly with time (Figure 5A). We used Western blotting to examine the expression of CA9 protein in the TE-2 cells. At the protein level, expression of CA9 increased with time under hypoxic but not normoxic conditions (Figure 5B). In CHEK-1 cells, the expression of CA9 protein did not increase under either normoxic or hypoxic conditions (data not shown). This confirmed that CA9 protein was induced by hypoxia. We also measured the expression of CA9 protein in the cell culture medium using ELISA and, interestingly, we found that CA9, which is a membrane protein, was present in the cell culture medium. The level of CA9 in the culture medium under hypoxic conditions was increased significantly when compared with that under normoxic conditions (*P*<0.01; Figure 5C).

#### Proliferation of ESCC cell lines under hypoxic conditions

We measured cell proliferation in two ESCC cell lines (TE-2 and TE-15), under hypoxic conditions, using the MTT assay. Each sample was measured three times. Both TE-2 and TE-15 cells proliferated significantly more under hypoxic than under normoxic conditions (*P*<0.01; Figure 6). In addition, the tendency for cell proliferation resembled a change of CA9 expression shown by ELISA.

## Discussion

We investigated the expression of CA9 in ESCC at both the protein and mRNA levels, and found that CA9 protein was expressed in tissue samples from 76 of 127 (59.8%) tumours. CA9, similar to HIF-1 (Pantuck *et al*, 2003), is a member of the hypoxia-induced pathway and is thought to be expressed specifically around the tumour centre, where hypoxic conditions prevail. We therefore performed CA9 scoring for three parts (tumour surface, centre and invasive front), but only the scores from the tumour centre were included in the statistical analyses. Our results reflected those obtained in studies of other solid tumours. Expression of CA9 has been reported in 48% of breast cancers (Chia *et al*, 2001), 79% of cervical cancers (Loncaster *et al*, 2001) and 81% of lung cancers (Swinson *et al*, 2003). However, in oesophageal cancer, many indicators of poor prognosis, such as Ki-67 and PCNA, which are cell proliferation markers, are expressed at the invasive front of the tumour. In this study, we found no significant correlation between CA9 expression at the tumour surface and invasive front and clinicopathological findings and prognosis (data not shown). In terms of IHC score, CA9 expression was significantly associated with tumour staging and poor prognosis. In other solid tumours, CA9 protein has been reported to be an independent factor related to poor prognosis (Chia *et al*, 2001; Loncaster *et al*, 2001; Brennan *et al*, 2006; Haapasalo *et al*, 2006; Lee *et al*, 2007). Driessen *et al* reported that CA9 expression was an independent prognostic marker in oesophageal cancers, especially adenocarcinomas and gastric cancer (Driessen *et al*, 2006), whereas in another study of oesophageal tumours, the degree of CA9 staining did not correlate with any of the pathological features examined (Turner *et al*, 1997). In our present study of ESCC, expression of CA9 protein was not independently related to poor prognosis. CA9 is a marker of hypoxia, and its expression is significantly correlated with tumour size. As a tumour grows in size, its centre gradually becomes starved of oxygen, and high expression of CA9 might therefore indicate that a tumour has a greater propensity for enlargement.

We studied the expression of CA9 mRNA in both normal and tumour tissues from 35 patients, using real-time RT–PCR. At the mRNA level, there was no significant correlation between CA9 expression and clinicopathological findings and prognosis (data not shown). In non-small-cell lung cancer, increased expression of CA9 mRNA in cancer tissues was significantly correlated with increased expression of the protein (Simi *et al*, 2006). However, in our study, we found no such correlation, perhaps because tissue samples were collected from the peripheral tumour areas, rather from the centre.

We confirmed *in vitro* that CA9 mRNA was expressed under hypoxic conditions in three ESCC cell lines, TE-2, TE-8 and TE-15, suggesting that upregulation of CA9 was controlled at the mRNA level. We also confirmed that CA9 was expressed at the protein level in these three ESCC cell lines under hypoxic conditions. Similar results have been reported for meningiomas (Yoo *et al*, 2007) and for several cell lines (Swinson *et al*, 2003; Robertson *et al*, 2004; Le *et al*, 2005). Comparison of the ESCC cell line TE-2 with an immortalised oesophageal cell line, CHEK-1, showed that expression of CA9 mRNA was induced in both under hypoxic conditions; however, the degree of CA9 expression differed greatly between the protein and the mRNA. This result suggests that CA9 might be induced in cells with higher malignant potential.

In this study, we also confirmed the presence of CA9 protein in the cell culture medium, a finding that has not been reported earlier. In ESCC cell lines, the level of CA9 in the culture medium was significantly increased under hypoxic conditions. CA9 is a membrane protein, and so it was very interesting to see that CA9 was present within the culture medium. It is unclear whether CA9 was secreted by the cancer cells or whether it was released from damaged cancer cells. In addition, we confirmed that oesophageal cancer cells under hypoxic conditions proliferated faster than cells under normoxic conditions, suggesting that CA9 has a role other than pH regulation alone. Robertson *et al* (2004) described that cells treated with CA9 interfering showed delayed growth under hypoxic conditions. In our study, cell proliferation and CA9 expression were induced under hypoxic conditions, suggesting that CA9 expression was correlated with cell proliferation.

In conclusion, our study has shown that hypoxia induces CA9 expression in ESCC and that this is related to poor prognosis. It has already been reported that (i) hypoxic conditions associated with tumours are related to resistance to chemotherapy and radiotherapy (Gray *et al*, 1953; Brizel *et al*, 1996; Hockel *et al*, 1996); (ii) low extracellular pH is a typical feature of the tumour microenvironment, which has an impact on cancer development (Svastová *et al*, 2004); and (iii) CA9 contributes to tumour growth and survival (Robertson *et al*, 2004). In addition, some ESCCs are relatively sensitive to chemotherapy and radiotherapy. Therefore, to improve the results of cancer therapy, it is important to control CA9, which is induced under hypoxic conditions and acidifies the tumour milieu. It is suggested that inhibition of CA9 may improve the effectiveness of chemotherapy and radiotherapy.

## Figures and Tables

**Figure 1:** Photomicrographs (magnification= × 200) of oesophageal squamous cell carcinoma and gastro-oesophageal junction immunohistochemically stained for carbonic anhydrase 9 (CA9). (**A**) The normal gastric mucosa was used as a positive control. The normal oesophageal mucosa was not stained for CA9; (**B**) weak staining in the tumour; (**C**) moderate staining in the tumour; (**D**) strong staining in the tumour.

**Figure 2:** Association of carbonic anhydrase 9 (CA9) tumour expression with outcome in 127 patients with oesophageal squamous cell carcinoma. Cancer-specific survival rates at 5 years after surgery were 66.5% for the CA9 low expression group and 33.3% for the CA9 high expression group. Kaplan–Meier curve is shown (*P*=0.0003, log-rank test).

**Figure 3:** Expression of CA9 mRNA in non-cancerous and cancer tissues from patients with oesophageal squamous cell carcinoma patients (*n*=35) assessed by real-time RT–PCR. Horizontal lines indicate mean values for each group. (N, non-cancerous tissue; T, cancer tissue) (*P*=0.0019, Mann–Whitney *U*-test).

**Figure 4:** Expression of CA9 mRNA assessed by RT–PCR in oesophageal squamous cell lines under normoxic and hypoxic conditions. Cell lines were cultured for 24 hours. Hypoxic conditions were generated with 1% O_2_ (N, normoxic; H, hypoxic).

**Figure 5:** *In vitro* assay for CA9 induced by hypoxia in an oesophageal squamous cell carcinoma line (TE-2) and in culture medium. (**A**) Comparison of CA9 mRNA expression in TE-2 cells and in the immortalised human oesophageal cell line (CHEK-1). CA9 expression was measured by real-time RT–PCR; (**B**) Expression of CA9 protein in TE-2 cells was measured by western blotting. Expression of CA9 protein was higher under hypoxic conditions; (**C**) Expression of CA9 protein in culture medium was significantly induced under hypoxic conditions (*P*<0.01). All examinations were done in triplicate. (N, normoxic; H, hypoxic).

**Figure 6:** Proliferation assay of oesophageal squamous cell carcinoma cell lines (TE-2 and TE15). (**A** and **B**) Both cell lines showed significantly greater proliferation under hypoxic than under normoxic conditions (*P*<0.01). All examinations were done in triplicate (N, normoxic; H, hypoxic).

**Table 1:** Correlations between clinicopathological characteristics and CA9 expression

		**CA9 (*n*=64)**	**CA9 (*n*=63)**	
**Parameters**	**Total (*n*=127)**	**Low**	**High**	***P*-value**
Age (mean±s.d.,^a^ years)	61.9±8.7	61.8±8.3	62.0±9.1	0.87^b^
				
*Gender*				0.0503^c^
Male	112	60	52	
Female	15	4	11	
Tumour size (mean±s.d.,^a^ cm^2^)	17.1±15.6	13.7±17	20.2±13	0.0235^b^
				
*Differentiation*				0.5429^c^
Well	29	12	17	
Moderate	66	35	31	
Poorly	32	17	15	
				
*TNM clinical classification pT (tumour depth)*				<0.0001^d^
T1	54	46	8	
T2	14	5	9	
T3	51	13	38	
T4	8	0	8	
				
*pN (regional lymph node metastasis)*				0.0031^c^
N0	57	37	20	
N1	70	27	43	
				
*pM (distant metastasis)*				0.0077^c^
M0	106	59	47	
M1	21	5	16	
				
*pStage*				<0.0001^d^
I	39	34	5	
II	36	16	20	
III	31	9	22	
IV	21	5	16	
				
*Location*				0.4777^c^
Upper	31	13	18	
Middle	79	48	36	
Lower	17	8	9	
				
*Lymphatic invasion*				0.0643^c^
Negative	40	25	15	
Positive	87	39	48	
				
*Blood vessel invasion*				0.006^c^
Negative	64	40	24	
Positive	63	24	39	

a s.d.

b Student's *t*-test.

c *χ*^2^ test.

d Fisher's exact test.

**Table 2:** Prognostic significance of CA9 expression and clinicopathologic parameters

**Risk factor**	**Reference factor**	***P*-value**	**Hazard ratio**	**95% CI** a
*Univariate*				
Age	62> *vs* 62<	0.1947	1.437	0.831–2.484
Histological grade	G1,G2 *vs* G3	0.0590	1.749	0.979–3.125
Primary tumour (T)	T1,T2 *vs* T3,T4	<0.0001	7.012	3.692–13.32
Regional lymph node metastasis (N)	Negative *vs* positive	<0.0001	7.697	3.462–17.11
Distant metastasis (M)	Negative *vs* positive	<0.0001	3.990	2.147–7.416
TNM stage (S)^b^	S1,S2 *vs* S3,S4	<0.0001	8.302	4.409–15.63
CA9 expression	Low *vs* high	0.0006	2.782	1.556–4.973
				
*Multivariate*				
Primary tumor (T)	T1,T2 *vs* T3,T4	0.0001	4.240	2.030–8.856
Regional lymph node metastasis (N)	Negative *vs* positive	0.0003	4.620	2.010–10.62
CA9 expression	Low *vs* high	0.7859	1.093	0.575–2.078

Cox proportional hazards analysis.

a Confidence interval.

b UICC (International Union Against Center) TNM classification.
